This article has been retracted.

# Analysis of Influencing Factors for Exercise Ventilation Efficiency of COPD Patients

**DOI:** 10.1155/2022/8376085

**Published:** 2022-08-29

**Authors:** Yu-mei Ge, Shan Nie, Nan Jia, Qiu-Fen Xu, Bo Xu, Hao-Yan Wang

**Affiliations:** Department of Respiratory Medicine, Beijing Friendship Hospital, Capital Medical University, Beijing, China

## Abstract

Dynamic pulmonary hyperinflation and abnormal air exchange are the primary causes of the exercise limitation of chronic obstructive pulmonary disease (COPD) patients. During exercise, COPD sufferers' lungs are dynamically hyperinflated. Increased inefficient ventilation reduces ventilation efficiency and causes a mismatch between ventilation volume and blood flow. The ventilatory equivalent for CO_2_ (VeqCO_2_) is a physiological parameter that can be measured using cardiopulmonary exercise testing. Therefore, the aim of this exploratory study was to perform cardiopulmonary exercise testing on people with COPD, investigate the impact of static pulmonary function on ventilation efficiency under the exercise state, and screen the predictive indicators of ventilation efficiency. *Subject*. The aim of this study was to look at the factors that influence the exercise ventilation efficiency of people with COPD. *Method*. A total of 76 people with COPD were recruited during the stable period. Age, gender, body height, body mass, and other basic information were recorded. The body mass index (BMI) was determined, and forced vital capacity (FVC), forced expiratory volume in one second (FEV1), residual volume/total lung capacity (RV/TLC), diffusing capacity of the lung for carbon monoxide (DLCO), and DLCO divided by the alveolar volume (DLCO/VA) were measured. The ventilatory equivalent for carbon dioxide (VE/VCO2) under the rest state (EqCO_2_rest), anaerobic threshold (EqCO_2_at), and maximum exercise state (EqCO_2_ max) were calculated to investigate the influencing factors for ventilation efficiency of people with COPD. *Results*. FEV1% was negatively correlated with EqCO_2_rest (*r* = −0.277, *P* value <0.05); FEV1/FVC % was negatively correlated with EqCO2rest and EqCO2at (*r* = −0.311, −0.287, *P* value <0.05); DLCO% was negatively correlated with EqCO_2_rest, EqCO_2_at, and EqCO_2_max (*r* = −0.408, −0.462, and −0.285, *P* value <0.05); DLCO/VA% was negatively correlated with EqCO_2_rest, EqCO_2_at, and EqCO_2_max (*r* = −0.390, −0.392, and −0.245, *P* value <0.05); RV/TLC was positively correlated with EqCO2rest and EqCO2at (*r* = 0.289, 0.258, *P*-value <0.05). The prediction equation from the multivariable regression analysis equation was *Y* = 40.04–0.075*X* (*Y* = EqCO_2_, *X* = DLCO/VA%). *Conclusions*. As the degree of ventilatory obstruction increased, the ventilation efficiency of the stable people with COPD under the exercise state showed a progressive decrease; the ventilation efficiency of the people with COPD decreased significantly under the maximum exercise state, and the ventilation capacity and diffusion capacity were the significant factors that affected the exercise ventilation efficiency. The diffusion function may predict the maximum ventilation efficiency and enable primary hospitals without exercise test equipment in developing countries to predict and screen patients at risk for current exercise based on limited information.

## 1. Introduction

Due to chronic airway limitation and poor pulmonary function, the cardiopulmonary exercise functions of people with COPD are aberrant. [1] However, studies have demonstrated that during exercise, the rate of decline in cardiopulmonary function is higher than the rate of progression of poor pulmonary function. [2] It is possible that it is linked to a decrease in inspiratory vital capacity and effective ventilation volume and abnormality of pulmonary air exchange caused by pulmonary hyperinflation. [3].

The ventilatory equivalent for CO_2_ (VeqCO_2_) is a physiological parameter that can be measured using cardiopulmonary exercise testing. According to previous research findings, people with COPD have significantly higher EqCO_2_ than people with normal lung function under the peak exercise state. It may be linked to the increase in physiological dead space volume/tidal volume (VD/VT) during exercise. [4] Studies have proved that it has low ventilation efficiency; that is, the rise in VE/VCO_2_ response during exercise is an independent predictor of the mortality rate in patients with chronic heart failure (CHF), pulmonary hypertension (PH), and chronic obstructive pulmonary disease (COPD). At present, there are few studies on the EqCO_2_ influencing factors, both at home and abroad. The goal of this study was to examine the factors that influence the ventilation efficiency of people with COPD in order to help primary care hospitals predict and screen patients at risk for exercise based on limited information.

## 2. Participants and Methods

### 2.1. Research Participants

From January 2016 to December 2019, 76 people with COPD who were receiving regular treatment during the stable period were recruited from the outpatients of Beijing Friendship Hospital's Respiratory Department. The study was carried out with the approval of the Beijing Friendship Hospital's Ethics Committee, and each participant provided written informed consent.

#### 2.1.1. Inclusion Criteria

(1) Diagnosed people with COPD: according to the GOLD Guidelines for COPD, [1] patients with dyspnea, chronic cough, or sputum expectoration and a history of exposure to COPD risk factors, having FEV1/FVC <70% after inhalation of bronchodilators and showing continuous airway limitation. (2) People with COPD during the stable period: the duration of the clinical stability was ≥6 weeks after the standardized treatment, that is, the drug treatment plan and drug dosage had not been changed due to changes in the patients' condition over the past 6 weeks. (3) The patients ranged in age from 40 to 85 years old. (4) The percutaneous oxygen saturation (SPO_2_) was >88% under the condition of inhalation of air under the rest state.

#### 2.1.2. Exclusion Criteria

(1) With a medical history of other pulmonary diseases, such as bronchiectasis (except for COPD complicated with bronchiectasis), interstitial lung disease, bronchial asthma, cystic fibrosis, infectious lung disease, thoracic deformity, and pneumonectomy, and without a history of respiratory tract infection over the past 6 weeks; (2) with severe cardiovascular diseases, such as acute left heart failure, malignant arrhythmia, uncontrolled hypertension, or with a medical history of the acute coronary syndrome within nearly one month; (3) with a medical history of major diseases of other systems, such as a malignant tumor, severe liver and kidney dysfunction, active autoimmune disease, lower limb bone and joint diseases that affect body activity, and limb activity disorder, cognitive disorder, and mental disorder caused by cerebrovascular diseases.

### 2.2. Research Methods

#### 2.2.1. General Data

Subjects were recruited, their genders and ages were recorded, body heights and body masses were measured, and the BMI [BMI = body mass (kg)/body height square (m^2^)] was calculated. Blood pressure, pulses, and SPO_2_ when inhaling air under the rest state were also measured. It was confirmed that the subjects had not been orally, intramuscularly, or intravenously treated with H1 receptor antagonists and adrenocortical hormone agents within 72 hours prior to the pulmonary function testing procedure, had not been treated with inhaled long-acting muscarinic antagonists (LAMA) and long-acting *β*_2_ receptor agonists/inhaled corticosteroids (LABA/ICS) within 24 hours prior to the pulmonary function testing procedure, and had not been treated with inhaled short-acting muscarinic antagonists (SAMA) and short-acting *β*_2_ receptor agonists/inhaled corticosteroids (SABA/ICS) within 4 hours prior to the pulmonary function testing procedure.

#### 2.2.2. Methods

All patients' static pulmonary functions (Master Screen Body, Care Fusion, Hochberg, Germany) were evaluated to determine the degree of airway restriction based on the GOLD stage and GOLD group.

The cardiopulmonary exercise testing (CPET) procedure was then carried out. The patients sat on an electronically braked cycle ergometer (ER 900L, Jaeger, Germany), which was equipped with an expiratory air collecting tube, an electrocardiograph, a blood pressure cuff, and an infrared blood oxygen saturation monitor. Their noses were clamped with a nose clip. The patients clenched their lips around the mouth bite. After 3 min of rest, the patients underwent 3 min of unloaded pedaling, followed by an incremental phase of exercise at a 10 W/min work rate. All participants were encouraged to cycle as long as they could until they were exhausted, then the load was reduced to a 20 W/min work rate, and the exercise was stopped after 4 to 6 minutes of slow exercise. Throughout the exercise test, the cardiopulmonary exercise tester (Oxycon Delta, JAEGER, Germany) was used to measure the parameters, such as oxygen uptake (VO_2_), carbon dioxide production (VCO_2_), and ventilation (VE), breath by breath. The anaerobic threshold (AT) was established via the V-slope method. According to the formula, EqCO_2_ = VE/VCO_2_, EqCO_2_rest, EqCO_2_at, and EqCO_2_max were calculated at rest, AT, and peak exercise. The direct measurement data were calculated based on the average value of 30 s measurement data.

#### 2.2.3. Statistical Processing

Data were analyzed using SPSS Statistics for Windows, Version 23.0. The normal distribution of data was confirmed using the Kolmogorov–Smirnov test. The results of the continuous variables were presented by mean and standard deviation, while the categorical variables were presented by percentage. The correlation analysis was assessed by the Pearson correlation coefficient. The screen influencing factors were analyzed using multiple linear regression (MLR). The results were considered statistically significant when the *P* value was <0.05.

## 3. Results

### 3.1. General Data

All 76 patients finished pulmonary function testing and CPET.

The anthropometric, functional characteristics of the objects were as shown in Table 1.

The characteristics of the cardiopulmonary exercise indicators of the test objects were as shown in Table 2.

### 3.2. EqCO_2_ Parameter Influencing Factors of People with COPD during the Stable Period

#### 3.2.1. General Influencing Factors

A correlation analysis was performed between the parameters EqCO_2_rest, EqCO_2_at, and EqCO_2_ max and age, body height, body mass, and BMI.  Table 3 shows the results: EqCO_2_at and EqCO_2_base were negatively correlated with BMI (*r* = −0.437, −0.308, *P* value <0.05), and EqCO_2_rest was positively correlated with body height (*r* = 0.274, *P* value <0.05).

#### 3.2.2. Pulmonary Function Influencing Factors

A correlation analysis was performed between the parameters EqCO_2_rest, EqCO_2_at, and EqCO_2_ max and the pulmonary function indicators FEV1, FEV1/FVC, RV/TLC, DLCO, DLCO/VA, RV, and VC-FVC. As shown in Table 4, FEV1% was negatively correlated with EqCO_2_rest (*r* = −0.277, *P* value <0.05); FEV1/FVC% was negatively correlated with EqCO_2_rest and EqCO_2_at (*r* = −0.311, −0.287, *P* value <0.05); DLCO% was negatively correlated with EqCO_2_rest, EqCO_2_at, and EqCO_2_max (*r* = −0.408, −0.462, −0.285, *P* value <0.05); DLCO/VA% was negatively correlated with EqCO_2_-rest, EqCO_2_at, and EqCO_2_max (*r* = −0.390, −0.392, −0.245, *P* value <0.05); RV/TLC was positively correlated with EqCO_2_rest and EqCO_2_at (*r* = 0.289, 0.258, *P* value <0.05).

In the group as a whole, there was a significant correlation of all pulmonary functions and EqCO_2_at, such as FEV1/FVC %, DLCO%, DLCO/VA%, and RV/TLC, except for FEV1%. Multivariable regression analysis revealed that the pulmonary function parameter DLCO/VA% was the only variable that significantly entered the regression as EqCO2at (Table 5). The prediction equation from the multivariable regression analysis equation was *Y* = 40.04–0.075*X* (*Y* = EqCO_2_, *X* = DLCO/VA%).

#### 3.2.3. Differences between Ventilation Efficiencies at Different Pulmonary Function Levels

Table 6 shows the differences between ventilation efficiencies at different pulmonary function levels. The numbers of cases at GOLD Level 1 and GOLD Level 4 were less than 10; therefore, the *t*-testing was only performed for GOLD Level 2 and GOLD Level 3.

## 4. Discussions

According to previous research findings, the subjective exertional dyspnea symptoms of people with COPD did not completely match the static pulmonary function indicators; clinical symptoms were not obvious, especially for mild and moderate patients; the decrease in pulmonary function was also not obvious under the rest state, but the patients' cardiopulmonary reserve functions significantly decreased. [5, 6].

CPET can play an important role in judging the severity of the disease, predicting survival time, identifying the cause of dyspnea, diagnosing complicated pulmonary vascular lesions, evaluating the treatment effect, and guiding pulmonary rehabilitation training. [7] Although CPET is not as valuable as conventional pulmonary function testing in the diagnosis of COPD, CPET is a sensitive method that can accurately quantify exercise tolerance. EqCO_2_ (ventilatory equivalent for carbon dioxide) is a critical parameter in the CPET, which is calculated using the equation: VeqCO_2_ = [V'_E_ − (*d*_syst_ × RR)]/V'_CO2_. EqCO_2_ was the focus of this study because previous research demonstrated that this parameter is most useful in the diagnosis of dysfunctional breathing [8]. The increase in EqCO_2_ indicates a decrease in ventilation efficiency [9, 10]. According to recent research, under the peak exercise state, the EqCO_2_ of people with COPD was significantly higher than that of people with normal lung function [10]. The reason can be correlated to an increase in the physiological dead space volume or tidal volume, which indicates a significant decrease in the ventilation efficiency of people with COPD [4]. Previous findings suggest that exercise ventilatory inefficiency is a physiological marker associated with clinically relevant end-points in patients with mild to end-stage COPD [11].

The previous research findings revealed that EqCO_2_rest, EqCO_2_at, and EqCO_2_max of people with COPD showed a progressive decline, while the EqCO_2_ of people with normal lung function hyperbolically decreased with increasing power during exercise. [12].

The research by Sun et al. [13] showed that for people with normal lung function, during the initial period of exercise, due to the hysteresis of nerve conduction, the increase in VE was relatively lower than that of VCO_2_, and EqCO_2_ was lower than that in the static state; when the exercise load increased to the point where the body began anaerobic glycolysis, intracellular bicarbonate neutralized lactic acid to produce a large amount of CO_2_, and chemoreceptors were excited, causing VE and EqCO_2_ to increase. Small airway obstruction and decreased compliance in people with COPD resulted in an increased residual air volume and thoracic expansion in the inspiratory state, limiting diaphragm function, shortening of inspiratory muscle fibers, and weakening of muscle strength; therefore, respiratory muscle fatigue was prone to occur during exercise. They have shown that reduced ventilatory efficiency during exercise is common in mild COPD, and this is primarily due to high physiological dead space (rather than alveolar hyperventilation or a relatively reduced tidal volume), resulting in a preponderance of lung units with high ventilation-perfusion ratios. [12] Because of the loss of gas exchange areas, increased dead space can reduce DLCO and KCO. We believe that the increase in EqCO_2_ is due to dead space rather than DLCO. We did not measure the dead space because artery blood was required.

Relevant studies revealed that the EqCO_2_ level of people with COPD was significantly higher than that of people with normal lung function under the high exercise state, which was correlated to an increase in the ratio between the physiological dead space volume and the tidal volume, indicating that the ventilation efficiency of people with COPD significantly decreased. [14] The research by Yuan and Wang [15] found that VE/VCO_2_ levels of people with COPD during the stable period progressively decreased at rest, AT, and peak exercise states, which was consistent with our findings.

Our study conducted a correlation analysis between multiple parameters of pulmonary function ventilation, diffusion, and VE/VCO_2_, demonstrating that for mild and moderate airway obstruction patients, ventilation efficiency at the AT state was clearly correlated with the degree of pulmonary function airway obstruction, diffusion function, and the ratio of the total residual. According to the GOLD classification, the greater the airway obstruction, the lower the ventilation efficiency, that is, the higher the VE/VCO2, indicating that the air exchange between people with COPD of varying severity had changed. [16] When the patient reached the maximum exercise state, ventilation efficiency was only correlated with the diffusion function and not with ventilation capacity. The most likely explanation is that after the anaerobic threshold, as exercise power increased, the body switched from aerobic metabolism to anaerobic metabolism, and the output of CO_2_ obviously increased, stimulating more VE and VCO_2_; furthermore, during exercise, the development of dynamic hyperinflation with a progressive increase in the end-expiratory lung volume (EELV) imposed additional elastic load on the ventilator system and was closely related to exertional dyspnea, and it, therefore, contributed to exercise limitation [17]. The ventilation efficiency calculated using VE/VCO_2_ was only correlated with the effective respiratory area, that is, the diffusion function but not with basic ventilation capacity under the rest state. Previous research proved that in patients who underwent lung volume reduction surgery, due to the improvement of alveolar ventilation, peak VE, VCO_2_, peak VE/VCO_2_, and other indicators were improved. [18, 19] The research on people with COPD based on exercise rehabilitation revealed that pulmonary rehabilitation has no significant effect on the improvement of ventilation efficiency in people with COPD. [20] This phenomenon also indirectly supported our research finding, that is, diffusion function is the only indicator of maximum ventilation efficiency, rather than ventilation and other indicators.

Alveolar ventilation and arterial blood gases PCO_2_ were used to adjust CO_2_ removal during exercise [21]. When the power was gradually increased, VE increased linearly with the increase in CO_2_ emissions within a considerable range of power. After the carbonic acid buffer period, the increase in VE was faster than that of VCO_2_ (an increase in the VE/VCO_2_ ratio). In our study, people with COPD did not exhibit the same ventilation characteristics at maximum exercise intensity as people with normal lung function under the maximum exercise state; that is, EqCO_2_ increased from the carbonic acid buffer period to the maximum exercise state. The probable reasons were that the people with COPD due to the increase in physiological dead cavities [14] had a ratio imbalance of ventilation volume and blood flow, and their VE/VCO_2_ was higher than that of people with normal lung function; furthermore, because of respiratory limitations caused by respiratory drive, respiratory muscle dysfunction, and other conditions, the VT of people with COPD could not be correspondingly increased according to the metabolic acidosis that occurred after the AT. EqCO_2_max was lower than EqCO_2_ during the period from *W*_at_ to *W*_max_. In addition to the aforementioned causes, it may also be due to the fact that the CPET examination is a test of self-control, COPD patients have poor exercise ability and reach MAX shortly after reaching AT, as indicated by the data, and *W*_max_ is similar to *W*_at_. At the same time, they may be afraid of unusual symptoms such as coughing and chest tightness and decide to skip the test.

The precise matching of alveolar ventilation with the metabolic rate during exercise is achieved by increasing minute ventilation. This increase is accomplished by increases in both the tidal volume and breathing frequency. During low-to-moderate intensity exercise, both tidal volume and breathing frequency increase roughly in proportion to exercise intensity [8], whereas at higher intensities, as our results showed that for COPD patients with a heavier GOLD grade, the expected ventilate ratio of maximum intensity exercise was lower. Therefore, due to the limitation of ventilatory function, it is necessary to rely more on the increased respiratory rate to meet metabolic requirements during certain intensity exercises.

Compared with the main ventilatory indicator of static lung function, diffusion function predicted decreased ventilatory efficiency during exercise (although it was not a particularly strong predictor). Although there are certain limitations to our study: the slope of VE/VCO_2_ indicates the efficiency of lung ventilation very well, EqCO_2_ is more convenient to obtain. Therefore, EqCO_2_ was selected for our research because it is more consistent with clinical practice. Due to the limited number of included GOLD1 and GOLD4 patients, the analysis of factors related to EqCO_2_ may not be clear, but based on existing data, the correlation between dispersion function indicators and EqCO_2_ has been shown. It may be possible for people who are difficult to implement CPET and institutions with limited medical conditions to screen people with hypoxia during exercise at an early stage and provide corresponding medical advice for the related risks.

## 5. Conclusion

In conclusion, the current study revealed the following trends: the ventilation efficiency of people with COPD during the stable period under the exercise state demonstrated a progressive decrease, and ventilation capacity and diffusion capacity were significant factors influencing ventilation efficiency. Among all lung function indicators, though not particularly strong predictors, the diffusion function may be able to predict the maximum ventilation efficiency.

Our study showed that DLCO/VA% was associated with EqCO_2_, which may be used as a means to screen hypoxia subjects during exercise, especially in primary hospitals without exercise test equipment, and implement relevant exercise prescriptions as early as possible.

## Figures and Tables

**Table 1:** Anthropometric, functional characteristics in COPD.

Items	Value(Mean ± SD)
Male/female	61/15
Age	64.35 ± 8.14
Body height (cm)	167.99 ± 7.68
Body weight (kg)	69.14 ± 13.82
BMI (kg/m^2^)	24.44 ± 4.29

*Static pulmonary function*	
FEV1%pred	59.41 ± 18.99
FEV1/FVC%	55.54 ± 11.77
RV/TLC	55.54 ± 12.13
DLCO%	59.88 ± 19.91
DLCO/VA%	76.60 ± 223.39

**Table 2:** CPET variables in COPD.

Items	Value
VO_2_max	1268.55 ± 289.12
VO_2_max/pred%	69.75 ± 13.89
Watts-at	60.21 ± 20.60
Watts-max	83.70 ± 25.72
Watts-max (W)	95.31 ± 26.3
HR-base	88.58 ± 11.85
HR-max	130.41 ± 18.77
HR-%	83.59 ± 10.96
VE-base	20.01 ± 5.37
VEmax	47.56 ± 12.08
VE%	58.30 ± 18.33
AT/(mL·min^−1^·kg^−1^) (*n* = 66)	13.05 ± 2.67
EqCO_2__rest_	36.63 ± 6.17
EqCO_2__at_	33.91 ± 5.21
EqCO_2__max_	33.04 ± 5.38

**Table 3:** Correlation of EqCO_2_ and anthropometric characteristics.

		BMI	Body height	Body weight	Age
EqCO_2_ at	Pearson correlation	−0.308^*∗*^	0.162	−0.214	0.246^*∗*^
	*P* value	0.012	0.194	0.085	0.046
	*n*	66	66	66	66

EqCO_2_ max^*∗*^	Pearson correlation	−0.185	0.113	−0.124	0.250^*∗*^
	*P* value	0.117	0.343	0.297	0.033
	*n*	73	73	73	73

EqCO_2_ rest	Pearson correlation	−0.437^*∗*^^*∗*^	0.271^*∗*^	−0.219	0.178
	*P* value	0.000	0.028	0.078	0.154
	*n*	66	66	66	66

^*∗*^significant difference, *P* < 0.05.

**Table 4:** Correlation of EqCO_2_ and key variables of pulmonary function.

		FEV1%	FEV1/FVC %	DLCO%	DLCO/VA%	RV/TLC
EqCO_2_rest	Pearson correlation	−0.277^*∗*^	−0.311^*∗*^	−0.408^*∗*^^*∗*^	−0.390^*∗*^^*∗*^	0.289^*∗*^
	*P*-value	0.024	0.011	0.001	0.002	0.023
	*n*	66	66	63	63	62

EqCO_2_at	Pearson correlation	−0.224	−0.287^*∗*^	−0.462^*∗*^^*∗*^	−0.392^*∗*^^*∗*^	0.258^*∗*^
	*P*-value	0.070	0.020	0.000	0.002	0.043
	*n*	66	66	63	63	62

EqCO_2_max ^*∗*^	Pearson correlation	−0.024	−0.086	−0.285^*∗*^	−0.245^*∗*^	0.095
	*P*-value	0.837	0.468	0.017	0.041	0.436
	*n*	73	73	70	70	69

^*∗*^significant difference, *P* < 0.05.

**Table 5:** Multiple linear regression with EqCO_2_ at as the dependent variable.

Coefficients						
Model		Unstandardized coefficients		Standardized coefficients	*t*	*P*
		B	Std. error	Beta		
1	(Constant)	40.040	2.387		16.771	0.000
	DLCO/VA%	−0.075	0.030	−0.321	−2.534	0.014

**Table 6:** EqCO_2_, RR, and VE at different exercise intensities by the GOLD stage.

	GOLD level 1	GOLD level 2	GOLD level 3	GOLD level 4	*t* value	*P* value
Number of cases	9	44	21	2		
EqCO_2_rest	32.33 ± 1.75	35.83 ± 1.02	39.64 ± 1.67	36.3 ± 2.26	−9.63	0.00
EqCO_2_at	29.46 ± 1.49	33.62 ± 0.87	35.58 ± 1.46	/	−5.68	0.00
EqCO_2_max	29.72 ± 1.32	32.99 ± 0.94	33.21 ± 1.39	29.05 ± 0.21	−0.657	0.51
RRrest	18.85 ± 5.31	21.95 ± 4.41	22.25 ± 5.94	23.5 ± 0.71	−0.38	0.71
RRat	24.86 ± 5.40	23.58 ± 3.66	26.70 ± 5.27	/	−2.26	0.03
RRmax	34.22 ± 7.43	31.05 ± 4.46	31.65 ± 6.02	30.0 ± 1.41	−0.52	0.61
%	79.7% ± 18,26	76.77 ± 16.56	76.38 ± 15.00	72.5 ± 3.54	0.02	0.98
VErest	15.71 ± 5.50	20.38 ± 5.51	20.31 ± 4.42	23.0 ± 5.66	0,10	0,92
VEat	28.30 ± 9.57	28.05 ± 8.07	31.31 ± 6.20	/	−1.32	0.19
VEmax	55.22 ± 9.24	48.61 ± 12.29	42.95 ± 10.09	32.5 ± 7.78	1.75	0.09
%	72.7 ± 14.97	60.15 ± 12.52	49.63 ± 10.76	36.5 ± 6.36	2.85	0.01

^*∗*^significant difference, *P* < 0.05.

## Data Availability

The data used to support the findings of this study are included within the article.

## References

[1] O’Donnell D. E., Lam M., Webb K. A. (1999). Spirometric correlates of improvement in exercise performance after anticholinergic therapy in chronic obstructive pulmonary disease. *American Journal of Respiratory and Critical Care Medicine*.

[2] Oga T., Nishimura K., Tsukino M., Sato S., Hajiro T., Mishima M. (2005). Exercise capacity deterioration in patients with COPD: longitudinal evaluation over 5 years. *Chest*.

[3] Stringer W., Marciniuk D. (2018). The role of cardiopulmonary exercise testing (CPET) in pulmonary rehabilitation (PR) of chronic obstructive pulmonary disease (COPD) patients. *COPD: Journal of Chronic Obstructive Pulmonary Disease*.

[4] Phillips D. B., Collins S. E., Stickland M. K. (2020). Measurement and interpretation of exercise ventilatory efficiency. *Frontiers in Physiology*.

[5] Murciano D., Ferretti A., Boczkowski J., Sleiman C., Fournier M., Milic-Emili J. (2000). Flow limitation and dynamic hyperinflation during exercise in COPD patients after single lung transplantation. *Chest*.

[6] Krol K., Morgan M. A., Khurana S. (2019). Pulmonary function testing and cardiopulmonary exercise testing: an overview. *Medical Clinics of North America*.

[7] Boutou A. K., Zafeiridis A., Pitsiou G., Dipla K., Kioumis I., Stanopoulos I. (2020). Cardiopulmonary exercise testing in chronic obstructive pulmonary disease: an update on its clinical value and applications. *Clinical Physiology and Functional Imaging*.

[8] Watson M., Ionescu M. F., Sylvester K., Fuld J. (2021). Minute ventilation/carbon dioxide production in patients with dysfunctional breathing. *European Respiratory Review*.

[9] Maekura R., Hiraga T., Miki K. (2014). Differences in physiological response to exercise in patients with different COPD severity. *Respiratory Care*.

[10] Caviedes I. R., Delgado I., Soto R. (2012). Ventilatory inefficiency as a limiting factor for exercise in patients with COPD. *Respiratory Care*.

[11] Neder J. A., Arbex F. F., Alencar M. C. N. (2015). Exercise ventilatory inefficiency in mild to end-stage COPD. *European Respiratory Journal*.

[12] Elbehairy A. F., Ciavaglia C. E., Webb K. A. (2015). Pulmonary gas exchange abnormalities in mild chronic obstructive pulmonary disease. Implications for dyspnea and exercise intolerance. *American Journal of Respiratory and Critical Care Medicine*.

[13] Sun X. G., Hansen J. E., Garatachea N., Storer T. W., Wasserman K. (2002). Ventilatory efficiency during exercise in healthy subjects. *American Journal of Respiratory and Critical Care Medicine*.

[14] Teopompi E., Tzani P., Aiello M. (2014). Ventilatory response to carbon dioxide output in subjects with congestive heart failure and in patients with COPD with comparable exercise capacity. *Respiratory Care*.

[15] Yuan W., Wang H. (2013). Correlation analysis of ventilation efficiency and exercise capacity of COPD patients. *Journal of Cardiovascular and Pulmonary Diseases*.

[16] Thirapatarapong W., Armstrong H. F., Thomashow B. M., Bartels M. N. (2013). Differences in gas exchange between severities of chronic obstructive pulmonary disease. *Respiratory Physiology and Neurobiology*.

[17] O’Donnell D. E., Webb K. A. (1993). Exertional breathlessness in patients with chronic airflow limitation: the role of lung hyperinflation. *American Review of Respiratory Disease*.

[18] Criner G. J., Belt P., Sternberg A. L. (2009). Effects of lung volume reduction surgery on gas exchange and breathing pattern during maximum exercise. *Chest*.

[19] Armstrong H. F., Dussault N. E., Thirapatarapong W., Lemieux R. S., Thomashow B. M., Bartels M. N. (2015). Ventilatory efficiency before and after lung volume reduction surgery. *Respiratory Care*.

[20] Laura de Araujo C., Araujo F. R. (2019). Pulmonary rehabilitation does not improve efficiency slopes in patients with COPD. *European Respiratory Journal. ERS International Congress abstract; European Respiratory Journal*.

[21] Stickland M. K., Butcher S. J., Marciniuk D. D., Bhutani M. (2012). Assessing exercise limitation using cardiopulmonary exercise testing. *Pulmonary Medicine*.

